This article has been retracted.

# Analysis of Enterprise Human Resources Demand Forecast Model Based on SOM Neural Network

**DOI:** 10.1155/2021/6596548

**Published:** 2021-06-21

**Authors:** Jiafeng Zheng, Ruijun Ma

**Affiliations:** ^1^Graduate School of Architecture, Planning and Preservation, Columbia University, New York, NY 10027, USA; ^2^School of Labor and Human Resources, Renmin University of China, Beijing 100872, China

## Abstract

Human resource planning is the prerequisite of human resource management, and the basic work of human resource planning is to predict human resource demand. Scientific and reasonable human resource demand forecasting results can provide important data support for enterprise human resource planning and strategic decision-making so that human resources management can play a better role in the realization of corporate goals. Because human resource demand is affected by many factors, there is a high degree of nonlinearity and uncertainty between each factor and personnel demand, as well as the incompleteness and inaccuracy of corporate human resource data. In this paper, the self-organizing feature mapping (SOM) artificial neural network prediction model is selected as the prediction model, and the input and output process of sample data is converted into the optimal solution process of the nonlinear function. In the application of the model, the human resource demand prediction index system is used as the input of the SOM neural network and the total number of employees in the enterprise is used as the output so that the problem of nonlinear fitting between human resource demand-influencing factors and human resource demand can be solved. Finally, through the empirical analysis of the enterprise, the model forecasting process is explained and the human resource demand forecast is realized.

## 1. Introduction

With the rapid development of the world economy, the demand for talents in various countries has become more and more urgent, and the talent reserve has become an important indicator of the comprehensive national strength of all countries in the world [1]. As we all know, compared with developed countries, our country is still at a significant disadvantage in the international talent competition. How to attract talents, retain talents, train talents, and formulate a human resource strategy that is in line with the current has become a compulsory course for the development and growth of enterprises [2]. Enterprise human resource planning is a kind of strategic planning. It is the behavior of an enterprise to predict the supply and demand of the required personnel in advance and to formulate a complete human resource strategy in order to achieve its predetermined goals and meet the needs of various personnel in the development process [3]. Scientific corporate human resources planning can provide important data support for the introduction of relevant human resource policies and the realization of corporate strategic goals.

Enterprise human resource forecasting consists of two parts: one is the forecast of human resource demand and the other is the forecast of human resource supply. Among them, the forecast of human resource demand is the prerequisite for the forecast of human resource supply. Only on the basis of clarifying the needs of personnel needed for future development according to their own actual conditions can the company predict the supply of human resources in a planned way and carry out reasonable human resource planning on the basis of the balance of supply and demand. Too many personnel demand forecasts will bring burdens to the enterprise, while too few personnel demand forecasts will cause a shortage of talents in the enterprise and hinder the further development of the enterprise. It can be seen that the human resource demand forecast is the basis of the corresponding operation plan in the human resource planning process. Self-Organizing Maps (SOM) [4] algorithm, as an unsupervised learning algorithm for clustering and high-dimensional visualization, is an artificial neural network developed by simulating the characteristics of signal processing by the human brain. This model was proposed in 1981 by Teuvo Kohonen, a professor at the University of Helsinki in Finland, and has now become the most widely used self-organizing neural network method. The WTA (Winner Takes All) competition mechanism reflects the most fundamental characteristics of self-organized learning [5].

Because human resource demand is affected by many factors, there is a high degree of nonlinearity and uncertainty between each factor and personnel demand, as well as the incompleteness and inaccuracy of corporate human resource data. This article chooses the SOM artificial neural network. The rest of the paper is organized as follows: Section 2 contains the literature review.  Section 3 contains the human resource demand forecast index system which is used as the input of the SOM neural network.  Section 4 contains the results which produce the total number of employees in the enterprise so that the problem of nonlinear fitting between the influencing factors of human resource demand and human resource demand can be solved.  Section 5 is the empirical analysis of enterprises; the model forecasting process is explained, which aims to provide enterprises with a more universally applicable, flexible, and accurate human resource demand forecasting method.

## 2. Related Works

There are qualitative and quantitative methods for human resource demand forecasting. At present, most of the forecasting methods in our country stay in qualitative forecasting research. Liu et al. [6] used the adaptive neural network optimal allocation model to realize the optimal allocation management of enterprise human resources. Jiang et al. [7] described in detail the application of the Delphi method in enterprise personnel prediction and pointed out that the method has high prediction accuracy. Son and Kim [8] have studied a large number of methods of enterprise personnel supply and demand forecasting, focusing on the analysis of manager replacement models, empirical forecasting methods, production function methods, and Markov models. Some scholars also use quantitative research methods to forecast human resource needs. Li et al. [9] used the linear regression method to predict the human resources status of an enterprise, but the method has poor adaptability. Once the prediction system is affected by an emergency, the prediction accuracy will be greatly reduced. Padhy et al. [10] analyzed four quantitative prediction models, namely, Markov model, nonlinear regression model, gray model, and neural network model. They pointed out that the gray prediction model and SOM neural network have high short-term prediction accuracy. The exponentially increasing data sequence has certain limitations in completing the personnel demand forecasting. Ahmad et al. [11] used the Markov model to predict the human resources of several companies. This method is convenient and efficient, but it has the problem of low accuracy of transition probability, which needs further improvement. Liu et al. [12] used the theory of a nonlinear dynamic system to predict the human resources of the enterprise and achieved good results, but the calculation process was cumbersome. Lee et al. [13] applied the support vector machine to the prediction of human resource structure and provided a new prediction method for human resource prediction. This method has been studied less at present and needs to be further studied.

Because the forecasting process is affected by many factors, a single forecasting model is not applicable. Therefore, many scholars have conducted in-depth research on the model combination. Zeng et al. [14] pointed out that the combination model is more accurate than the single model for human resource prediction. Kang et al. [15] obtained a new combination model by the weighted average of the two forecasting models. However, the correlation between the models and the different usage premises will have a certain impact on its prediction effect. Jeong et al. [16] elaborated on the development history and existing problems of combined forecasting technology and studied a variety of combined forecasting methods. At the same time, there is a high nonlinear mapping relationship between various influencing factors and personnel requirements, especially when the external environment changes greatly. Then, the selection of key indicators has become one of the important issues of human resource forecasting. Kumar et al. [17] summarized the superiority of the gray relational analysis method in the selection of nonlinear indicators.

At present, there are many qualitative and quantitative forecasting methods used in the forecasting of enterprise personnel demand, such as the Delphi method, regression analysis method, trend extrapolation method, and other methods that are relatively mature in foreign applications. However, these methods have not yet been popularized in our country. Demand forecasting mostly stays on qualitative analysis. In addition, the enterprises do not pay attention to the collection of historical data of enterprises and the nonlinear relationship between the results of human resource demand index forecasts in their own development process. The existing methods cannot reasonably predict the human resource needs of enterprises, so this article constructs a method for human resource demand forecasting suitable for enterprises.

## 3. SOM Neural Network

There are many text clustering algorithms. Among them, the SOM clustering algorithm based on Self-Organizing Mapping is a particularly suitable method for clustering large-scale documents. The SOM clustering algorithm was first proposed by Finn Kohonen in 1982. It is an unsupervised training neural network. The process of white organization is actually unsupervised learning. It uses white body training, and white motion clusters the input patterns.

### 3.1. Basic Principles of SOM

The network structure of SOM is shown in Figure 1. It consists of an input layer and a competition layer (output layer). The number of neurons in the input layer is *n*, and the competition layer consists of a one-dimensional or two-dimensional planar array of *m* neurons. The network is fully connected, that is, each input node is connected to all output nodes.

The SOM network can map any dimensional input pattern into a one-dimensional or two-dimensional graph in the output layer, and keep its topological structure unchanged; through repeated learning of the input pattern, the network can make the weight vector space and the probability distribution of the input pattern converge [18], that is, probability retention. Each neuron in the competition layer of the network competes for the response opportunity to the input pattern, and the weights related to the winning neuron are adjusted in a direction that is more conducive to its competition. That is, the winning neuron is the center of the circle, and the neighboring neurons are excited side feedback; while showing inhibitory side feedback to the neurons in the distant neighbors, the neighbors stimulate each other, and the distant neighbors inhibit each other. Generally speaking, the nearest neighbor refers to the neuron whose radius is about 50 *μ*m∼500 *μ*m from the neuron that sends a signal; the far neighbor refers to the neuron whose radius is about 200 *μ*m∼2 mm. Neurons farther than the distant neighbors exhibit weak excitation, as shown in Figure 2. Because the curve of this interaction is similar to the hat worn by the Mexicans, it is also called the “Mexican hat.”

### 3.2. Process of the SOM Algorithm

The specific process of the SOM algorithm is as follows:

(1) Assign a small random initial value to the weight *w*_*ij*_; set a larger initial neighborhood *R*, and set the network cycle number *K*.
(2) Given a new input mode *x*_*i*_: *X*_*i*_={*x*_1_, *x*_2_,…, *x*_*n*_}, input it to the network.
(3) Calculate the distance *s*_*i*_ between mode *x*_*i*_ and all output neurons, and select the neuron *c* with the smallest distance from *x*_*i*_, namely,
  (1) $$\begin{array}{c} \text{Inf}\left\{s_{ij}\right\}=x_{i}-w_{ij}. \end{array}$$
Then, *j* is the winning neuron.
(4) Update the connection weight of node *j* and its domain node:
  (2) $$\begin{array}{c} w_{ij}\left(k+1\right)=\frac{x_{i}-\left(\lambda \left(k\right)-1\right)w_{ij}\left(k\right)}{\lambda \left(k\right)}, \end{array}$$
where *λ*(*k*) ∈ (0, *∞*) is the gain function which gradually decreases with time.
(5) Select another learning mode to provide to the input layer of the network, and return to step (3) until all input modes are provided to the network.
(6) Let *k*=*k*+1 and return to step (2), until *k*=*K*.

In the learning of the Self-Organizing Mapping model, *K* ∈ [5000,10000] is usually taken.*R* gradually decreases as the number of learning increases. The gain function *λ*(*k*) ∈ (0, *∞*) is also the learning rate. Since the learning rate *λ*(*k*) gradually tends to zero with the increase of time, it is guaranteed that the learning process must be convergent. General requirements are

(3) $$\begin{array}{c} \sum_{i}^{n}\lambda \left(k\right)⟶\infty ,\\ \sum_{i}^{n}\lambda^{2}\left(k+i\right)\leq \infty . \end{array}$$

Among them, *λ*(*k*+*i*) ∈ (0, *∞*),  *i*=1,2,…, *∞*. In the actual weight coefficient self-organization process, generally, for a continuous system, take *λ*(*k*)=*k*.

For discrete systems, then take *λ*(*k*+*i*)=*k*+*i*.

### 3.3. Limitations of the SOM Algorithm

The development of unsupervised learning is still immature, and the SOM algorithm still has some limitations [19–22] as follows:

1. The network structure is fixed and cannot be changed dynamically
2. During network training, some neurons can never win and become “dead neurons”
3. The SOM network cannot add new categories before complete relearning
4. When the input data is small, the training result usually depends on the sample
5. The initial state of the network connection right and the parameter selection in the algorithm have a greater impact on the convergence performance of the network

For this reason, some scholars have proposed different improved algorithms to overcome these shortcomings to varying degrees from different aspects. The specific process of the SOM algorithm is shown in Figure 3.

## 4. Theoretical Framework of Enterprise Human Resource Demand Forecasting System

The human resource demand forecasting system solves the problems that need to be analyzed when forecasting human resource demand, the content of the forecast, and the use of forecasting models; that is, it provides the technical preparation work required before the forecast and the technical means used in the forecast. Through the analysis of the constituent elements of the predictive model construction subsystem and the characteristics of human resource demand forecasting, reasonable constituent elements are provided for the construction of the model. The forecasting system provides a systematic theoretical guidance framework for human resource demand forecasting. The framework diagram is shown in Figure 4.

### 4.1. Construction of the Preliminary Selection Index System for Human Resource Demand Prediction Based on SOM Neural Network

There are many commonly used methods of primary selection index mining, such as the Delphi method and target hierarchy method [23–25]. In order to have an intuitive understanding of the principles and advantages and disadvantages of various methods, it is convenient to choose a method suitable for the construction of the primary selection index system for human resource needs. Changes in the internal and external environment of the enterprise bring about changes in personnel needs. As time changes, demand-influencing factors will also change accordingly. In order to select indicators that affect human resource demand more comprehensively and flexibly, this article uses the existing human resource demand-influencing factors as the basis to further add and delete the existing indicator system.

The first-level indicators in this paper are constructed from the perspective of resource matching, which means that human resource needs are matched with corporate financial resources, material resources, market resources, corporate human resources, and corporate strategy. The development level of an enterprise affects the demand for its personnel, and the number of resources invested determines the level of development of the enterprise. Therefore, the investment of resources by an enterprise is the decisive factor for the needs of enterprise personnel. Only by ensuring the coordination and matching of various resources in the development process of an enterprise can it better promote the realization of the enterprise's strategic goals and realize the efficient and optimized development of the enterprise.

#### 4.1.1. Human Resources Horizontal Matching Perspective

From this perspective, it mainly examines the matching of human resources and financial resources, material resources, and market resources. The main purpose of corporate financial resources is to realize the normal production and operation of the enterprise and the strategic planning of the enterprise, to allocate the financial resources of the enterprise, that is, to invest and finance the enterprise. Investment generally revolves around two directions: one is scientific and technological activities and the other is production and operation activities. The investment behavior of an enterprise will cause changes in the production activities of the enterprise, which requires the participation of matching human resources. Therefore, the capital investment in the production research and development is selected as a secondary indicator for matching human resource requirements with corporate financial resources. The three-level indicators under this indicator can be the ratio of corporate R&D investment and the added value of corporate fixed assets. Enterprise material resources refer to the plant, equipment, land, production materials, and other material resources used to support the normal production and operation of the enterprise. The increase in the material resources of the enterprise or the change in the conditions of technical equipment will have an impact on the demand for enterprise personnel [26–28]. Therefore, the supporting conditions of enterprise development are selected as the secondary index for matching human resources and enterprise material resources, and the choice of the third-level indicator needs to be determined according to the actual material support situation of the enterprise. Enterprise market resources are an important factor in measuring the development space of an enterprise. In order to facilitate the measurability of indicators, market demand is selected as another secondary indicator. If the market demand is large, the company's future demand for personnel will increase accordingly. The three-level indicators of market demand investigation are mainly measured by factors such as the total number of customers.

#### 4.1.2. The Perspective of Vertical Matching of Human Resources

The perspective of vertical matching of human resources mainly examines the matching of human resources needs and human resources' own conditions. The labor cost trends, labor productivity, and personnel mobility of an enterprise will all have an impact on the demand for employees. Here, these three items are selected as secondary indicators. Among them, the labor cost trend is mainly reflected by the wage level of the company, and the flow of personnel is measured by indicators such as promotion, resignation, and retirement.

#### 4.1.3. The Perspective of Matching Human Resources with Corporate Strategy

The strategic goals of an enterprise can be divided into two parts: economic indicators and growth indicators. Economic indicators are financial indicators. Although they cannot fully reflect the implementation effects of corporate strategies, they are easy to quantify and facilitate statistical analysis. Many noneconomic indicators will eventually be reflected indirectly through economic indicators. Therefore, this article chooses the economic measurement indicators of corporate strategy. Production demand and enterprise scale are two important measurement indicators that reflect the realization of corporate strategy: production demand is mainly measured by the total output value of the enterprise and sales indicators. The sales indicators are sales, sales volume, and sales profits. In order to avoid crossover between indicators, the number of enterprise assets is selected as the three-level indicator of enterprise scale. The former starts from the ownership of the company, the latter starts from the ownership, and the liabilities are included in the value of the company.

Based on the above analysis, construct a secondary index system for human resource demand forecasting as shown in Table 1.

What needs to be explained is that the indicators that affect human resource demand forecasting in different industries and even at different stages of the development of the same enterprise will change. Enterprises should appropriately eliminate and add new ones based on the secondary indicator system according to the current actual situation which adapts to the current demand forecast index system.

### 4.2. Design of the SOM Neural Network Model Based on Human Resource Demand Forecast

SOM neural network has the characteristics of nonlinear mapping ability, fault tolerance, self-learning ability, and so forth. Therefore, SOM neural network has strong applicability in human resource demand forecasting. The following will analyze the reasons why the SOM neural network has these characteristics and explain its modeling process. The information processing system of the artificial neural network is established with reference to the reaction process of the biological nervous system. Imitating the structure of the biological nervous system and the information processing process, the establishment of an artificial neural network requires three key elements: the mathematical model of the neuron, the topological structure of the neural network, and the training and learning algorithm of the neural network.

The determination of the neural network structure mainly includes three parts: the determination of the number of hidden layers and the number of nodes; the determination of the number of neurons in the input layer; and the determination of the number of neurons in the output layer.

1. Determination of the number of hidden layers and the number of nodes: the number of hidden layers and the number of nodes affect the prediction accuracy of the SOM neural network. In 1989, Robert Hecht-Nielson proved that any three-layer neural network containing only one hidden layer can complete the nonlinear mapping from *h* dimension to *k* dimension. The neural network model with only one hidden layer has low prediction accuracy. In order to improve the accuracy of prediction, measures can be taken to increase the number of hidden layers or increase the number of nodes in each hidden layer, but at the same time, this will also make the neural network change. It is more complicated and increases the training time of the network connection weight coefficient. Generally speaking, it is necessary to adjust the number of hidden layers and the number of nodes in the network training process according to the actual situation, until the global error is minimized. Based on the high prediction accuracy of model construction and the simplicity of model construction, it is determined that, in human resource demand forecasting, the number of hidden layers is determined to be 1-2, and the number of nodes needs to be determined according to specific examples.
2. Determination of the number of neurons in the input layer: generally speaking, the number of neurons in the input layer is known when the SOM neural network is applied. When forecasting human resource demand, the number of neurons in the input layer is the number of indicators for human resource demand forecasting. According to the index system constructed before this article, the number of input neurons for a specific company has several key indicators.
3. Determination of the number of neurons in the output layer: in this article, the output of the SOM neural network is the total human resource demand of the enterprise, so the number of neurons in the output layer is 1.

## 5. Application of the SOM Neural Network Model

In order to explain the applicable conditions, forecasting process, and forecasting accuracy of each model in the combined forecasting system constructed by the SOM neural network, this paper selects a company to show the forecasting process of the model, and its total human resource demand from 2018 to 2020 is forecasted.

### 5.1. Establishment and Determination of the Enterprise Index System

First, a three-level indicator system should be constructed based on the framework of the second-level indicator system and combined with the actual situation of the enterprise. Secondly, use the gray correlation method to screen the three-level indicators and determine the key indicators that affect the human resource needs of the power supply enterprise. The construction of the index system needs to comprehensively consider the aspects of production and R&D capital investment, enterprise development support conditions, market demand, labor productivity, and enterprise scale that affect human resource demand from the matching perspective mentioned before. However, according to the principle of the specific analysis of specific issues, the influencing factors are the same for different companies. This article refers to the inspection indicators of the superior company on the company and combines the company's own operating conditions to construct a human resource demand forecast index system that meets the company's needs, as shown in Table 2.

### 5.2. Key Indicator Screening

After the indicator system is constructed, it is necessary to screen out the key indicators that have a greater impact on human resource requirements, as shown in Figure 5. Through the introduction of the previous article, this paper chooses the method of calculating the comprehensive correlation degree in the gray correlation method to screen the key indicators.

Then, sort the degree of relevance; the greater the degree of relevance, the greater the impact on personnel needs. The ranking shows that the number of customers, the length of transmission lines, the number of electricity sold, and the number of substations have a greater impact on personnel requirements. Therefore, these four indicators are selected as the key indicators that affect the personnel needs of enterprises to predict the total number of future personnel.

### 5.3. SOM Neural Network Prediction Implementation

The prediction process of the SOM neural network is divided into two steps: one is to use the optimization model to predict the key indicator data in 2020 and the other is to use historical data to train the SOM neural network to imitate the key indicator prediction value as the SOM neural network after the training is completed input to predict the total demand for corporate personnel from 2018 to 2020. Use the historical data of key indicators to use the optimization model to predict the indicator data from 2018 to 2020. The predicted values are shown in Figure 6.

### 5.4. Network Training and Simulation

After predicting the indicator data gray, start to train the SOM neural network. Before training, the data needs to be normalized to ensure that all data are at the same magnitude to improve the efficiency of training. After normalization, the network parameters should be defined. Here, the training target is set to 0.00001, the maximum number of training times is 50,000, and the learning rate is set to 0.01. Then, use the data from 2010 to 2017 for network training, and the data from 2018 for simulation.

The linear regression method is used to compare the actual output value with the expected output value. The result shows that the actual output value has a good tracking effect on the expected output value, the calculated *R* = 0.9999, and the training effect is better. The linear regression of the actual output and expected output of the SOM neural network and the standard error is shown in Figures 7 and 8.

Next, use the historical data in 2020 to simulate the model. The actual output value in 2020 is 6270, and the calculated relative error is 1.1820%, which is less than 3%, which has a good simulation effect. After the network training simulation is completed, the 2018–2020 index data can be used as the model input to predict the company's total staff demand for 2018–2020. The forecast results are shown in Figure 9.

## 6. Conclusions

Based on the research of relevant literature, this article conducts an in-depth analysis of the applicability, advantages, and disadvantages of existing human resource demand forecasting methods and points out that each method has its specific limitations for the characteristics of human resource demand forecasting. On this basis, the applicability of the SOM neural network model in human resource demand forecasting is analyzed, and an index system for human resource demand forecasting is constructed. And based on the analysis of the selected dimensions of the forecasting method, a human resource demand forecasting system is constructed. Finally, use a company to verify the prediction process and accuracy of the SOM neural network model. Through simulation prediction, it shows that the model has strong applicability and high prediction accuracy. At the same time, the company's total personnel demand for the next three years is predicted. The analysis results show that the model has strong applicability when the number of employees in an enterprise increases or decreases rapidly.

## Figures and Tables

**Figure 1:** SOM network structure.

**Figure 2:** Neuron interaction mode.

**Figure 3:** The specific process of the SOM clustering algorithm.

**Figure 4:** Human resource demand forecasting system diagram.

**Figure 5:** Plot of historical data of indicators.

**Figure 6:** SOM model predicted values of key indicators.

**Figure 7:** Error of SOM neural network.

**Figure 8:** Linear regression of SOM neural network.

**Figure 9:** SOM neural network prediction results.

**Table 1:** List of secondary indicators.

First-level indicators	Second-level indicators
Corporate financial resources	Production R&D capital investment

Enterprise material resources	Enterprise development support conditions

Enterprise market resources	Market demand

Human resources	Labor cost trends
	Labor productivity
	The flow of personnel

Corporate strategy	Corporate scale
	Production demand

**Table 2:** Enterprise index system.

First-level indicators	Second-level indicators	Third-level indicators
Enterprise material resources	Enterprise development support conditions	Transmission line length
		Number of substations

Enterprise market resources	Market demand	Total customers
		Power supply population

Corporate strategy	Corporate scale	Total assets
	Production demand	Electricity sales

## Data Availability

The data used to support the findings of this study are available from the corresponding author upon request.
